# Observation of Visual Quality after Femtosecond Laser-Assisted Cataract Surgery Combined with Trifocal Intraocular Lens Implantation

**DOI:** 10.1155/2022/1519416

**Published:** 2022-07-01

**Authors:** Jianli Ma, Xuequan Sun, Yang Liu, Yumei Liu

**Affiliations:** ^1^Department of Ophthalmology, Zhengda Guangming Eye Group, Weifang Eye Hospital, Shandong 261000, China; ^2^Department of Ophthalmology, Chongqing Wanzhou Aier Sunshine Eye Hospital, Wanzhou Chongqing 404100, China

## Abstract

**Objective:**

This study is the first observation of Alcon's PanOptix trifocal intraocular lens (IOL) implanted in 55 cataract patients with femtosecond laser-assisted cataract surgery.

**Methods:**

Fifty-five patients (63 eyes) with cataract were treated with femtosecond laser-assisted cataract surgery combined with trifocal IOL implantation. Visual acuity, defocus curve, higher order aberration (HOA), refractive stability, eyeglass removal rate, and satisfaction were evaluated and analyzed.

**Results:**

We found that the visual acuity of patients with near, intermediate, and distance vision was better than 0.1 LogMAR at 1, 3, and 6 months after the completion of surgery. The uncorrected near visual acuity (UCNVA), uncorrected intermediate visual acuity (UCIVA), and uncorrected distance visual acuity (UCDVA) of patients at 1, 3, and 6 months after surgery were compared with those before operation, showing statistical significance. Six months after the operation, all patients' surgical eyes had a smooth transition in the defocus range from +0D to -2.5D, and the visual acuity of the surgical eyes reached a level better than 0.1 LogMAR. The statistical results of 6-month follow-up showed that the eyeglass removal rate at near, intermediate, and far distances was 100%. At 6 months postoperatively, only 1 case had nocturnal glare, which affected life; 3 cases developed glare and halo but did not affect life. The patient satisfaction rate was 98.18%.

**Conclusions:**

Femtosecond laser-assisted cataract surgery with trifocal IOL implantation can remove the lens from the patient with satisfactory visual quality and significantly improve the postoperative satisfaction of the patient.

## 1. Introduction

Cataract, one of the most important blinding diseases in the world [1], is caused by various reasons, such as aging, genetic immunity, radiation injury, and other causes of lens metabolism disorders and protein denaturation, which makes the lens cloudy and the turbid lens block light from entering the retina, resulting in blurred vision [2]. At present, surgery is the main method to treat cataract [3]. In the earliest stage, the treatment is mainly to break the suspensory ligament around the lens, dislocate the lens, and sink into the vitreous cavity, so that light could enter the eye [4]. However, this method can only temporarily solve the problem, as the patient will be in a state equivalent to high myopia when refraction is lost after lens dislocation [5]. The sinking of the lens into the vitreous cavity is more likely to cause inflammation and eventually loss of vision [6].

At present, phacoemulsification (PHACO) is the mainstay of treatment for cataract among various surgical treatments [7]. PHACO works by inserting a PHACO probe through a small incision made in the cornea or sclera, crushing the lens nucleus into a chylous shape using high-frequency vibration. The chylous is systematically sucked out, keeping the anterior chamber full, and then an intraocular lens (IOL) is implanted [8]. PHACO is an ideal cataract surgery with small incision, no pain, short operation time, and not obvious postoperative astigmatism [9]. However, the operation is costly and difficult to master, and it is still difficult to completely replace other methods [10]. Therefore, it is of great significance to find a more effective treatment that can facilitate recovery. Femtosecond laser-assisted surgery, on the other hand, is a surgical procedure within the scope of PHACO technology, which is carried out by the computer according to the set program, with high stability and accurate cutting [11, 12]. However, there are still few reports investigating its therapeutic effect in cataracts.

The procedure involves removing the damaged lens, which is often replaced with a new artificial lens to restore vision [13]. An IOL is an artificial lens made from a synthetic material that can replace the lens and has been developed for six generations [14]. The original monofocal IOL cannot be adjusted by the ciliary muscle and the zonules as normal lenses do nor can it be adjusted to a certain range of focal length [15]. Bifocal IOL uses the refraction and diffraction principle of light to form the near and far focus, which relatively improves near vision, but has the problem of reduced contrast sensitivity [16]. Furthermore, the trifocal IOL also adopts the diffraction principle, but with optimized and improved structure to further improve the near and far vision [17]. However, there are few reports about femtosecond laser-assisted cataract surgery with trifocal IOL implantation in China. In this study, 53 cases (63 eyes) of cataract patients implanted with AcrySof® PanOptix® IOL were studied and analyzed for their clinical effects, so as to provide reference value for the extensive development of Focus IOL.

## 2. Materials and Methods

### 2.1. Research Participants

The study has been approved by the Ethics Committee of our hospital. Fifty-five patients (63 eyes) with cataract admitted to our hospital from November 2018 to November 2019 and met the surgical requirements were included. Inclusion criteria are as follows: (1) lens opacity; (2) patients with visual acuity <0.3; (3) regular corneal astigmatism ≤0.75D; and (4) Alpha angle <0.5 mm and Kappa angle <0.3 mm. Exclusion criteria are as follows: (1) severe corneal opacity, obstructing the passage of laser; (2) unable to cooperate with this study; (3) severe systemic diseases (such as diabetes); and (4) other eye diseases, such as macular degeneration. All patients in this study signed an informed consent form and agreed to a 6-month follow-up visit. General information of subjects is shown in Table 1.

### 2.2. Preoperative Examination

Patients all underwent routine eye examinations before treatment, including eye B-ultrasound, slit lamp microscope, corneal endothelium, optical coherence tomography, best-corrected visual acuity (BCVA), and uncorrected visual acuity (UCVA). IOL was measured by an IOLMaster optical biometer. The power of IOL was calculated by SRK/T formula, and the target diopter was set close to 0°.

### 2.3. Surgical Methods

All operations were performed by the same experienced doctor. The pupils were fully dilated before the operation, and the surgical eye of the patient placed in the supine position was subjected to topical anesthesia. LenSx (Alcon, America, Figure 1(a)), a femtosecond laser-assisted cataract surgery system, was used to make a 2.2-mm main membrane incision at the 120° axial position of the cornea and a 1.2-mm lateral corneal incision at the 20° axial position. The diameter of the femtosecond laser anterior capsule incision was 5.3 mm. After presplit nucleus treatment, the patient was transferred to the PHACO operating room. Following routine disinfection, the eyelid organs of the patient were opened, and viscoelastic agent was injected into the anterior chamber. After removing the free anterior capsule membrane with capsulorhexis forceps, the nucleus and cortex of lens were aspirated using an ophthalmic PHACO instrument (Shanghai Jumu Medical Instrument Co., Ltd., Figure 1(b)), the remaining cortex was fully injected and polished, and then the capsule was implanted into AcrySof® PanOptix® IOL (Alcon, Fort Worth, TX, USA), Figure 1(c)). The viscoelastic agent in the capsule was completely sucked out, and the anterior chamber was formed with the mouth closed. After the operation, we applied topical Bishu eye ointment and bandaged the operated eyes. AcrySof® PanOptix® IOL is a single aspheric IOL. The main body and support part were made of hydrophilic acrylic material with hydrophobic surface characteristics. The front surface was designed with a combination of refraction and diffraction, with an optical diameter of 6 mm, a maximum diameter of 11 mm, a short distance of 33d, a medium distance of 1.66d, a central 4.34 mm area with trifocal design, and a bifocal design for the surrounding area.

### 2.4. Postoperative Follow-Up and Observation Indexes

At 1, 3, and 6 months after surgery, the following postoperative detection indexes of patients were collected through medical records inquiries and telephone visits.

#### 2.4.1. Vision Test

Uncorrected near visual acuity (UCNVA), uncorrected intermediate visual acuity (UCIVA), and uncorrected distance visual acuity (UCDVA) were measured before and 1, 3, and 6 months after operation. UCNVA was detected with standard near vision chart, and the detection distance was 40 cm. UCIVA was tested using the standard near vision chart, and the detection distance was 80 cm. And UCDVA was evaluated using the standard logarithmic visual acuity chart, with the detection distance of 40 m.

#### 2.4.2. Defocus Curve Measurement

Six months postoperatively, the comprehensive refractometer was used to reduce the spherical degree from +2D to -4D with 0.5d as the first gear, and the corresponding spherical degree vision of the patient was detected. The defocus curve was drawn with visual acuity as *Y*-axis and spherical degree as *X*-axis.

#### 2.4.3. Higher Order Aberration

The higher order aberration (HOA) was measured with an I-Trace visual function analyzer (Shanghai Hanfei Medical Instrument Co., Ltd.) with a pupil diameter of 3 mm. The total HOA, Trefoil, Coma, and Spherical aberration were recorded before operation and 1, 3, and 6 months after operation. All tests were completed by a doctor who is skilled in operating the system, instructing the patient to open both eyes and open the fixation target. The average was taken after three measurements.

#### 2.4.4. Refractive Stability

Six months after the operation, the diopters (D) of the patients were observed and recorded, and the spherical equivalent (SE) of D was calculated. The histogram was drawn according to the interval distribution of ±1.0d, ±0.75D, ±0.50D, and ±0.25D.

#### 2.4.5. Eyeglass Removal Rate and Satisfaction

Six months after surgery, the subjective visual quality of patients was investigated with the self-made questionnaire, including the rate of eyeglass removal and visual satisfaction. The postoperative eyeglass removal rate was assessed from UCNVA (watching mobile phone), UCIVA (reading), and UCDVA (watching TV). Visual satisfaction, evaluated according to halo, glare, and other visual interference phenomena, was divided into 4 grades ranging from dissatisfied to very satisfied.

### 2.5. Statistical Methods

SPSS 23.0 statistical software (IBM SPSS, Inc., Chicago, IL, USA) was used to statistically analyze the data. Qualitative data were expressed as *n* (%), and quantitative data were expressed as (^−^*x* ± *s*). Qualitative data, quantitative data, and repeated measurement data were analyzed by *χ*^2^, *t*-test, and analysis of variance (ANOVA), respectively. *P* < 0.05 means the difference is statistically significant.

## 3. Results and Discussion

### 3.1. Comparison of Preoperative and Postoperative Visual Acuity

At 1, 3, and 6 months after the operation, the near, intermediate, and distance vision of patients were found to be better than 0.1 LogMAR. UCNVA, UCIVA, and UCDVA at 1, 3, and 6 months after surgery were compared with those before surgery, and significant differences were determined (*P* < 0.05), while the comparison of UCNVA, UCIVA, and UCDVA at 1, 3, and 6 months after surgery revealed no statistical significance among different postoperative periods (*P* > 0.05, Figure 2).

### 3.2. Defocus Curve after Surgery

After the operation, we followed up all the patients for 6 months and found that all the operated eyes of patients had a smooth transition in the defocus range of +0D to -2.5D, with a visual acuity level better than 0.1 LogMAR (Figure 3).

### 3.3. Comparison of HOA before and after Surgery

The HOA, trefoil aberration, coma aberration, and spherical aberration of patients 1, 3, and 6 months postoperatively were compared with those before the operation, and significant differences were determined (*P* < 0.05), while the HOA, trefoil aberration, coma aberration, and spherical aberration showed no statistical significance among different postoperative periods (1, 3, and 6 months after surgery) (*P* > 0.05, Figure 4).

### 3.4. Postoperative Refractive Stability Distribution of Patients

During the 6-month follow-up, we found that 63.49% of the affected eyes had SE within ±0.25D, 87.30% had SE within ±0.50D, 96.83% had SE within ±0.75D, and 100.00% had SE within ±1.00D (Figure 5).

### 3.5. The Eyeglass Removal Rate and Satisfaction of Patients

We followed up the patients for 6 months after surgery and calculated to find that the eyeglass removal rate at the near, middle, and long distances was 100%. During the follow-up, only 1 patient was reported with night glare, which affected life, and 3 cases experienced glare and halo that did not affect life. The patient's satisfaction rate was 98.18% (Figure 6).

## 4. Discussion

Cataracts can be divided into congenital cataracts and acquired cataracts. The former, also known as developmental cataracts, exists in the embryonic period and is mostly caused by genetic metabolic diseases, while the latter is attributed to the patient's own diseases, metabolic abnormalities, poisoning, trauma, etc. The pathogenesis of cataract is mainly crystal protein degeneration, oxidative stress, and lens epithelial cell (LEC) apoptosis [18]. The lens transmits light, which is projected onto the retina to produce vision. Lens proteins, which play an important role in maintaining lens transparency, come in two main types: water-soluble and insoluble. Water-soluble proteins are dominant, but when insoluble proteins begin to increase due to various reasons, the water-soluble ones will decrease accordingly, forming an uneven medium and light scattering that affects the light transmittance and light refraction ability of the lens, which is the basis for the onset of cataracts [19]. There are three main types of water-soluble proteins: *α*, *β*, and *γ*. The *α*-crystallin molecular chaperone active peptide can inhibit the production of insoluble proteins. Changes in the structure or quantity of *β*/*γ*-crystallin protein will alter the lens structure and produce insoluble proteins. Therefore, lens protein denaturation is to provide a material basis for the occurrence of cataracts [20]. The production of 8-hydroxyguanine, which is produced in deoxyribonucleic acid (DNA), disturbs the base pairing and causes changes in protein function. DNA single-strand breaks are also one of the factors in the formation of cataracts, and LEC apoptosis is the cytological basis [21].

LenSx is mainly based on the principle of photolysis and dielectric breakdown. It uses high irradiance, high-precision focusing, and short pulse laser spot to be highly localized in transparent tissues (such as cornea), so that the beam can be absorbed in a very short time. At 100°C to 300°C, the energy generates plasma, whose expansion and contraction generates shock waves. While the expansion and contraction of tissues leads to cavitation and formation of bubbles that fuse and burst to allow accurate cutting of adjacent tissues [22]. When this technology is applied to the cornea and lens, bubbles are generated only at the specified depth within the lens due to the wavelength (1053 nm) not being absorbed by corneal tissue and anterior lens capsule, which can evaporate the tissue in the micron-level plane.

In the development of IOL, monofocal IOL solves the problem of blindness that may occur after lens removal. However, because its lens can only be used as a lens to replace its refractive function, it is still necessary to wear glasses to adjust the vision after monofocal IOL implantation, so as to basically restore normal vision. The lens adjusts its thickness through the human body to adjust the focus, but the IOL can only obviously fix its size, and the implantation of it cannot use the principle of natural lens to adjust the focus. Therefore, bifocal IOLs were invented based on the principle of refraction and diffractive optics to adjust the focus. According to different principles, bifocal IOLs are divided into refractive, diffractive, and hybrid IOLs. The refractive IOL is a refracted light with aspherical concentric rings on its front surface to produce near and distance vision. The diffractive bifocal IOL uses the principle of light wave dynamics to construct diffraction steps and diffraction zones of the micro slope ring on the back surface to produce near and distance vision. The hybrid IOL is designed to achieve diffraction in the middle and refraction in the periphery. The width and height of the annulus are gradually changed from the center to the periphery to smooth out the light and thus achieve clear vision in the near and far. However, the disadvantage of these designs is that nonfocal imaging on the focal plane can also appear blurred, which will interfere with focus imaging, presenting as glare and halos, decreased contrast sensitivity, and loss of fine vision [23]. To solve these problems, a trifocal IOL was developed.

At present, trifocal IOLs include Fine Vision trifocal IOLs, Zeiss trifocal (AT LISA tri839MP) IOLs, and PanOptix trifocal IOLs. Fine Vision trifocal IOLs are developed based on the principle of diffraction, with the diffraction ring highly focused on myopia and intermediate vision, allowing for near vision increase by +3.5D and intermediate vision increase by +1.75D. The pupil size adjusts the light to enter to adjust distance vision, with 43% of the light used for distance vision, 28% for near vision, and 15% for intermediate vision [24]. AT LISA tri839MP IOLs are based on the design of aspheric refraction and diffraction. Optically, it is divided into two parts, namely, the trifocal area in the middle and the traditional bifocal area in the periphery, which can compensate +3.33D near vision and +1.66D intermediate vision [25]. The above two trifocal IOLs have achieved good results in clinical applications, but their astigmatism problems cannot be ignored.

PanOptix trifocal IOLs, which are the latest AcrySof series developed by Alcon Corporation of the United States in 2015, were used in this study. The optical diameter of such IOLs is 6.0 mm, and the total diameter is 13.00 mm, with 15 diffraction zones in the optical zone, which can distribute the light energy to 3 focal points. Among them, the energy of the first diffracted class is redistributed to the zero, second, and third classes. The zero class is used for distance vision to retain the original single focus lens vision, the second class is used for vision, increasing +2.17D, and the third class is used for near vision, increasing the near vision by +3.25D [26]. The results of this study show that patients can obtain good vision better than 0.1 LogMAR in near, intermediate, and far vision at 1, 3, and 6 months after surgery, with well-recovered UCNVA, UCIVA, and UCDVA. Compared with the research results of the AT LISA tri 839MP IOL implantation by Kretz et al. [27], the application effect in this study is more ideal and stable.

The defocus curve is an important indicator evaluating the performance of multifocal IOLs, which mainly reflects the continuous visual range of patients [28]. The changes in vision are reflected by measuring the visual performance of patients at different distances. The change in distance is mainly due to the change of the lens to cause defocus, so it is called the defocus curve. The abscissa of the defocus curve is the power of the added lens, and the ordinate is the visual acuity. The 6-month postoperative defocus curve of this study showed two peaks at 0D and -2.5D, but the transition was smooth in the middle, and the visual acuity level of the surgical eye was better than 0.1 LogMAR. The two peaks indicate that the patient's distance and near vision are sufficiently clear after the operation, and the gentle change indicates that the far-near conversion is stable and clear. This is mainly because the PanOptix trifocal IOL increased +2.17D vision and increased +3.25D near vision, which is consistent with the findings of Poyales et al. [29].

Studies have pointed out that nonfocal imaging on the focal plane can also be blurred and interfere with focal imaging due to HOA. The glare and halo, decreased contrast sensitivity, and loss of fine vision after the above-mentioned bifocal IOL are due to HOA [30]. Measuring the total HOA of the trifocal IOL helps to reflect the objective changes in visual quality. This study found that the total HOA, coma aberration, spherical aberration, and clover aberration of the whole eye at each postoperative period were significantly lower than those before surgery, similar to the research results of Zein El-Dein et al. [31]. Therefore, the HOA in this study is not high, and the patients can obtain a more satisfactory visual quality.

Refractive stability reflects the performance of cataract surgery [32]. If the refractive stability is good, it means high-accuracy cutting during the operation will not damage the cornea and other tissues. In our study, 63.49% of the affected eyes had SE within ±0.25D, 87.30% had SE within ±0.50D, 96.83% had SE within ±0.75D, and 100.00% had SE within ±1.00D. It demonstrates the accuracy of LenSx and the advantages of small tissue damage, without damaging the cornea, iris, and other capsule tissues of the lens, which also provides an effective location for subsequent IOL implantation. Donmez et al. [33] reported that PanOptix trifocal toric IOL has excellent refractive stability and can provide excellent visual quality for patients.

Patient satisfaction and eyeglass removal rate reflect the patient's overall surgery and postoperative recovery. In this study, the eyeglass removal rate of near, middle, and far distances was 100%. Six months after the operation, only 1 patient was reported with night glare, which affected life, and 3 cases experienced glare and halo that did not affect life. The patient's satisfaction rate reached 98.18%, which is relatively high. The results of the above complications and satisfaction rate were similar to those of Brozkova et al. [34]. Kretz et al. [27] also pointed out in their study that the surgical satisfaction rate of patients under trifocal IOL (AT LISA tri 839MP) intervention was 80%, which was significantly lower than that of 98.18% in this study.

The novelty of this study lies in the analysis of femtosecond laser-assisted cataract surgery combined with trifocal IOL implantation from the perspectives of visual acuity, defocus curve, HOA, refractive stability, eyeglass removal rate, and patient satisfaction. It is confirmed that femtosecond laser-assisted cataract surgery combined with trifocal IOL implantation has a positive effect on the visual quality of cataract patients and can provide comfortable visual perceptions for patients. However, this study still has several limitations. First, it is a small single-center study, which may have information collection bias. Second, the subjects included in this study were mainly middle-aged and elderly patients. If the study on young patients can be increased, it will be beneficial to further verify the effectiveness of femtosecond laser-assisted cataract surgery combined with trifocal IOL implantation in young patients. Third, the effect of this therapy on patients' contrast sensitivity and defocus curve has not been analyzed. In the future, the research project will be gradually improved around the above points.

This study, as far as we know, presents the first observation of Alcon's PanOptix trifocal IOL implanted in 55 cataract patients with femtosecond laser-assisted cataract surgery and studied and analyzed its clinical effects, providing valuable references for the wide development of trifocal IOLs. Femtosecond laser-assisted PHACO combined with trifocal IOL implantation has achieved good application effects in the treatment of cataract patients. It can provide natural full-course vision and quick recovery for patients, with small trauma, few side effects, high postoperative stability, and high patient satisfaction after surgery.

## Figures and Tables

**Figure 1:** (a) Femtosecond laser. (b) Phacoemulsifier for ophthalmology. (c) Alcon's PanOptix trifocal IOL.

**Figure 2:** Comparison of patients' visual acuity before and after surgery. Note: ∗ indicates *P* < 0.05 compared with before treatment.

**Figure 3:** Defocus curve after trifocal IOL implantation.

**Figure 4:** Comparison of HOA before and after surgery. Note: ∗ indicates *P* < 0.05 compared with before treatment.

**Figure 5:** Postoperative refractive stability distribution of patients.

**Figure 6:** The eyeglass removal rate and satisfaction of patients.

**Table 1:** General information of subjects.

Number of cases (*n*)	Operative eye (*n*)	Male (*n*)	Female (*n*)	Age (^−^*x* ± *s*, years)	Astigmatism (^−^*x* ± *s*, D)
55	63	21	34	57.94 ± 8.41	0.34 ± 0.17

## Data Availability

The labeled dataset used to support the findings of this study are available from the corresponding author upon request.
